The article "Construction and Application of Curriculum System of Design Major Integrating Environmental Protection and Big Data" was published in 2022. Journal: J Environ Public Health.

# Construction and Application of Curriculum System of Design Major Integrating Environmental Protection and Big Data

**DOI:** 10.1155/2022/7496172

**Published:** 2022-09-12

**Authors:** Yan Kou

**Affiliations:** NanYang Vocational College of Agriculture, School of Arts and Humanities, Nanyang, Henan 473000, China

## Abstract

Design subject curriculum system is a major subject in the field of design education. The gap between ideal and reality makes the design of the curriculum system of design discipline a serious and urgent problem. Facing the “integration of industrialization and industrialization,” we can explore the professional curriculum system of environmental design and construction. And the method of constructing the corresponding system is initially proposed. The fuzzy comprehensive evaluation method is used to evaluate and analyze the comprehensive effect of the model. According to the suggestions of experts and teachers, the designed indicators include 4 first-level indicators and 16 corresponding second-level indicators. The primary indicators include classroom response, teacher satisfaction, teaching effectiveness, and teaching environment. According to the fuzzy comprehensive evaluation steps and corresponding calculation methods, the final evaluation results are obtained.

## 1. Introduction

The “14th Five-Year Plan” period will be a critical period for national industrial transformation and upgrading. Design major exists as a creative and cultural industry and is regarded as an important tool to promote industrial upgrading. It can promote the transformation of the cultural and creative industry to high-end comprehensive design services, and promote the extension of the design service field and the upgrading of service models [1]. Design majors should actively adapt to the needs of local economic and social development and cultural industry innovation. It not only needs to combine its own school-running orientation, service orientation, and subject characteristics, but also clarify the training objectives, training norms, and curriculum for professional talent system. The purpose of environmental art design in the 21st century is to use science and technology to integrate art, humanities, and nature. In this way, a living space with high cultural taste and in line with human nature can be created. With the high development of China's social economy, people's quality of life has gradually improved, the level of material civilization and spiritual civilization has continued to improve, and the requirements for environmental art design have also continued to increase. At the same time, environmental art design is still a very young and new discipline in China [2]. Although it is developing rapidly and urgently needs a large number of specialized talents in environmental art design, there is a serious shortage of design talents with high cultural accomplishment and professional technical level in this young industry. Thus, higher education in Chinese environmental art design is born. Departments of architecture and fine arts in major universities in China have established environmental art design majors to meet the needs of social development for high-quality intelligent and compound design talents. They have also actively carried out the teaching reform of environmental art and design to accelerate the training of high-level professionals in environmental art and design [3–5].

At the same time, people's living environment starts from the needs of people. It constitutes an environmental system with more complex functions, more diverse types, and richer forms. Due to the increasingly close interaction between people and the environment, people's awareness of environmental protection is increasing. At the same time, the status of art participating in environmental transformation is also becoming more and more prominent. “Environmental art,” which is difficult to find in classical aesthetics in the past, comes into being. Then, it develops into a relatively independent art design category that integrates multidisciplinary knowledge. It makes people begin to explore the harmonious relationship between the environment and people from the height of culture and art. It also endows human environmental construction activities with more sustainable and better vitality [6]. In 1988, the former Central Academy of Arts and Crafts changes the major of interior design to the major of environmental art design, and expands the content of interior design to outdoor environment design. Subsequently, colleges and universities across the country have established this major [7]. Under the circumstances of reform and opening up and the rapid development of economic construction at that time, in order to meet the needs of urban construction for outdoor environmental design in a timely manner, the establishment of the environmental art design major greatly meets the requirements of the development of the times. Since the establishment of the environmental art design major, the number of Chinese colleges and universities offering this major has gradually increased in the past ten years. At the same time, the number of students graduating from environmental art and design is also increasing every year. And the proportion of students engaged in this industry is also increasing day by day, as shown in Figure 1.

The era of big data has come, but the curriculum system of environmental design talent training schools rarely involves the courses of big data design. There are certain problems in the adjustment and integration of the curriculum system. This paper takes the construction of the curriculum system of environmental design major as the research object. Its purpose is to investigate the current state of the curriculum system of environmental design majors. On the basis of discovering the deficiencies in the course system construction of environmental design and exploring the existing problems in the course system construction process, the corresponding construction strategies are put forward. By trying to build a curriculum system that meets the requirements of smart tourism development, it will lay a solid foundation for the future tourism industry to cultivate qualified talents and provide a strong guarantee for the career development of students [8].

The research significance of this paper mainly includes the following points.

### 1.1. Theoretical Significance

Through the research on the existing curriculum system of environmental design, the key ability of talent demand in the era of big data is analyzed. By finding out the deficiencies of the existing curriculum system, it stimulates the renewal of the curriculum system construction concept of environmental design and promotes the innovation of the curriculum system design concept.

### 1.2. Practical Significance

The practical significance has the following three aspects:

1. It is necessary to attract the attention of the school of environmental design to the curriculum system. Through the reflection of various problems existing in the construction of professional curriculum system, the construction of curriculum system is improved.
2. It is necessary to attract the attention of education administrative departments and secondary vocational tourism colleges and universities to the construction of the curriculum system of secondary vocational tourism management. Thereby, it provides a guarantee for the improvement of the quality of students in secondary vocational tourism colleges and the promotion of their careers.
3. It is necessary to attract the attention of the academic circles to the construction of the curriculum system of the vocational tourism management major. By promoting its gradual improvement, the perfect combination of industry needs and talent training has been achieved.

## 2. Related Theories

### 2.1. Definition of Big Data

The term Big Data was first coined by McKinsey in the book The Third Wave, but it does not give a complete definition of Big Data. In 2011, a McKinsey Global Institute research report defined big data as a collection of data larger than traditional databases can collect, store, and analyze. Wikipedia defines big data as the amount of data involved. And it cannot be manually acquired, managed, and processed into human-readable information within a reasonable time. Some scholars believe that big data is a powerful tool that generates, collects, or stores a huge amount of data and can be used to make smarter decisions. They also believe that big data is a collection of data that is processed by using advanced data storage, management, analysis, and visualization technologies. Big data is characterized by large capacity, various types, fast access speed, and low-value density. At the same time, it is rapidly developing into a new generation of information technology and services. It is possible to discover new knowledge and create new value by collecting, storing, and correlating data from scattered sources and various types of data [9].

Big data needs to be used as a tool. This will not confuse the concepts of big data and big data analysis techniques. Big data analysis technology is a technical means of using big data. It can discover new knowledge and new value from data. Thinking of big data as an asset is primarily an abstract description of the value of big data. Big data is composed of massive amounts of data. Based on big data analysis technology, the collected massive data is cleaned, desensitized, processed, and calculated. It not only obtains potential and regular information and knowledge, but also realizes the functions of prediction and judgment[10].

The integration of big data and the curriculum system of design majors is the general trend of education development. The professional curriculum system in the era of big data integrates several advantages and fully reflects the development characteristics of its informatization. The details are shown in Figure 2.

Figure 2 shows the characteristics of the professional curriculum system in the big data environment. The relatively important ones of all the features include real-time data, reliable decision-making, and intelligent interaction. The data runs through the professional curriculum system, and teachers can obtain real-time student learning data and give feedback on the classroom situation. According to the feedback of the professional curriculum system data, teachers can timely make teaching strategies and make decisions that are based and reliable. Teaching in the environment of professional curriculum system, teachers and students through remote control, can well reflect the intelligence of teacher-student interaction [11, 12].

### 2.2. Curriculum and Its System

In school education, curriculum refers to the process of learning subject content. But after the twentieth century, under the influence of Dewey and other progressive curriculum ideas, curriculum scholars begin to redefine the concept of curriculum. People from different perspectives have different opinions on the definition of “reshaping” the curriculum, criticizing, modifying, and replacing the original meaning of the curriculum. According to the statistics of American scholar Brewer, the term curriculum has at least one meaning. This gives the curriculum diverse and even esoteric meanings [13]. The definition of a course with a large audience is nothing more than limiting its connotation from the following dimensions.

### 2.3. Curriculum Structure

Curriculum system refers to the whole formed by some interrelated and restrained things. Therefore, the system is not a single thing. It contains a number of things that are related to each other. The system contains the meaning of the system to a certain extent. It also reflects the characteristics of integrity. China's curriculum system can also be divided into broad and narrow perspectives [14].

From a narrow perspective, the curriculum system refers to the internal structure of each course and the way each course is combined. The curriculum structure is the curriculum system. Both of them are equivalent. The meaning is that the courses offered by the school have different divisions of labor and cooperate with each other. It is the most important part of the teaching plan [15].

From a broad perspective, the so-called curriculum system refers to the basic principles of specific educational concepts and values. It is a combination of many elements that make up the curriculum in a certain way. In turn, these elements can better promote the smooth realization of the goals of the curriculum system.

The courses are divided vertically and can be divided into 3 levels:

1. Macro level: it refers to the establishment of disciplines and majors in colleges and universities.
2. Meso-level: it refers to how to arrange the course content of a specific major and how to design the course structure.
3. Micro level: it refers to how to arrange and determine the teaching content of a certain course in a certain major.

### 2.4. Element Analysis of the Curriculum System

The horizontal analysis of the curriculum shows that the curriculum is composed of multiple links. Each link is independent of each other, and each has different content and characteristics, but each link affects and restrains each other [16]. Whether the goals and functions of the curriculum system, as shown in Figure 3, can be realized depends on whether each link is normal. At the same time, it also depends on whether the cooperation between each link is good. The author will elaborate and analyze the components of the curriculum system in detail.

#### 2.4.1. Course Targets

Curriculum objectives refer to the specific goals to be achieved by the curriculum itself. It is the degree to which students at a certain educational stage are expected to develop morality, intelligence, and physique. Subject area curriculum objectives relate to the expected requirements for student growth and development in a particular discipline in a particular area. It should have a strong disciplinary nature and fully reflect the characteristics of the discipline itself. This is the commonly understood course goal.

The course objectives have the following characteristics:

1. The course goal reflects the characteristics of finality, but it also reflects a certain process.
2. The course goal should be a complete system. It reflects the school's overall and unified planning for teaching work and student education.
3. Curriculum objectives need to provide direction for educational activities. The entire teaching of the school is based on this and revolves around this goal.

#### 2.4.2. Course Content

The so-called curriculum content refers to the teaching content of various majors and disciplines offered by the school. It can refer not only to the specific content of a certain discipline, but also to all the content of all disciplines under a certain major, and it can also refer to the sum of all the content of all disciplines offered by the school. Curriculum content occupies a central position in the curriculum structure, which reflects and embodies curriculum objectives. Colleges and universities will be affected by cultural factors, ideological factors, student factors and other factors when selecting and determining course content. Different people will have different views on the nature of the course. This makes a big difference in their understanding and perspective of course content.

#### 2.4.3. Course Structure

The characteristics of the course structure are as follows:

1. The curriculum structure needs to proceed from an objective basis. The curriculum structure is an artificial structure and not an unnatural structure in nature. It is the result set by people according to certain curriculum principles, and it must have certain objective basis.
2. The curriculum structure reflects the characteristics of orderliness.
3. The so-called order refers to the relationship between the elements and parts of things according to certain rules and mutual transformation. The orderliness of the curriculum structure means that the various elements and parts that constitute the curriculum structure interact with each other according to certain rules. It is embodied in the dual order in space and time.
4. The curriculum structure has the characteristics of sequential change.
5. Specifically, the curriculum structure should be able to adapt to the changing needs of society and students, and the curriculum should be able to change constantly. It is necessary to proceed from the social reality and according to the new situation and new needs, through continuous adjustment of the curriculum structure to make it more reasonable.

#### 2.4.4. Curriculum Implementation

Domestic scholars have made different definitions of the concept of curriculum implementation. Curriculum implementation can be seen as the process of putting the curriculum plan into practice. Taking curriculum implementation as one of the links in curriculum development and preparation, it is considered that curriculum implementation is the process of implementing curriculum plans. The concept of curriculum implementation as part of curriculum change is a process that requires putting innovation into practice. At present, it has become the leading understanding of “curriculum implementation” at home and abroad.

#### 2.4.5. Course Evaluation

Curriculum evaluation refers to educational evaluation. By systematically collecting certain information and according to certain value standards, it can judge the development and changes of educated people in educational activities. At the same time, to what extent the factors that constitute its change meet the needs of social and individual development. It can provide the basis for the self-improvement of the evaluators and the scientific decision-making of the relevant departments. Curriculum evaluation in a narrow sense that refers to the activity or process of judging the value of curriculum plans and curriculum standards in improving students' learning. It generally includes core content such as course objectives and course plans. The range of subjects for course evaluation is very wide. A representative view holds that the object of curriculum evaluation has at least one aspect: curriculum design, curriculum used by teachers, student achievement, and curriculum system.

## 3. Current Situation of the Curriculum System of Environmental Design Major in Colleges and Universities

### 3.1. Profile Analysis

The history of setting up environmental protection design majors in Chinese colleges and universities is not long. At present, most of this major is offered in art colleges and some engineering colleges. Due to the different understanding and understanding of the concept of environmental protection and the different nature and foundation of schools, there are differences in the positioning of professional construction and the setting of teaching content. The status quo is that the environmental design major with comprehensive discipline characteristics is only positioned in a single direction of interior design.

Although some are called environmental design majors, the curriculum is only the content of interior design. There are also schools that focus on landscaping such as interior decoration and decoration. The reason for the formation of this situation is the problem of academic cognition. It is also the need for social development in a specific historical period. At the 21st century, social development needs will be different. The students who are trained away from the teaching system based on architecture are too narrow in their professional scope and have a single knowledge structure. Due to the lack of comprehensive quality of students and poor social adaptability, this state is contrary to the needs of national construction for talents with a comprehensive knowledge structure. Therefore, through reforming the professional structure of environmental art design and carrying out discipline construction, the task of cultivating high-quality intelligent and compound design talents has been placed in front of the education department. With the development of society, from the perspective of industry construction and management, it is necessary to establish a construction and design talent pattern with three levels of relationship: urban planning and design, architectural design, and environmental art design. The emerging discipline of environmental design has the characteristics of pluralistic structure. It is a systematic project that scientifically and holistically grasps disciplines such as urban planning, architecture, art, and gardening. It has the dual nature of art and technology. The requirements for environmental art designers are comprehensive quality and the ability to organize and collaborate. In urban construction, it plays an important role in improving the quality of the environment.

According to the survey, practitioners believe that the abilities that they need to have are mainly as follows. The survey results show that 12.13% of the people give top priority to their overall quality and ability to organize and collaborate. The proportion of people who put the ability to work independently first is 26.32%. The proportion of people who put professional skills and operational ability first is 15.69%. The proportion of people who put professionalism and initiative in the first place is 8.96%. The proportion of people who put interpersonal communication and teamwork spirit first is 36.9%. The relationship between the ability of the above survey results and the proportion of supporters is shown in Figure 4.

### 3.2. Problems Existing in the Design Major Integrating Environmental Protection

#### 3.2.1. Lack of Knowledge about the Design Industry

The prosperity of the design industry has made the society and parents pay unprecedented attention to design. This kind of attention not only promotes the development of design education, but also raises people's irrational expectations for the design industry. This has caused art and design education to expand rapidly when its foundation is not yet solid. Not only are colleges and universities rushing forward in response to the market orientation, but many secondary vocational and technical schools also offer relevant design courses. However, there is a lack of teachers and theoretical research, which will inevitably cause the quality of education to be difficult to guarantee. At the same time, society's understanding of design is also too simplistic. It is generally believed that with the foundation of art and software operation, design work can be carried out.

#### 3.2.2. The Training Objectives Do Not Meet the Employment Needs of the Enterprise

The training goal of the original curriculum system of the existing design major is to imitate the foreign training system and be highly professional. As a result, graduates cannot reach the level of designers. Such graduates do not meet the recruitment requirements of employers who are not only familiar with basic knowledge of graphic design and software operations, but also can integrate environmental protection and big data features. Employers need the breadth of knowledge and proficient operational and practical ability, but also the depth of knowledge and research significance.

#### 3.2.3. The Curriculum System Lacks Scientific Planning

Course objectives tend to focus only on the techniques and methods in the creation. The emphasis on the cultivation of students' thinking and creativity is neglected. It also ignores the research on the internal relationship between courses and the logic of their own development. The content of the course is too fragmented. The teaching of basic courses often becomes a simple patchwork of teaching content. It is difficult to link the subject content with the spirit of the times. It has deviated from the basic principles of applying what has been learned.

Due to the weak research on curriculum and teaching issues, the subject-systematized curriculum model is a fixed model under specific conditions in the early stage of industrialization. In the context of the information age, it has finally become an immutable teaching routine. The curriculum and teaching plan have not been properly adapted to the market, social development, and new technology development system, and the mechanism has not been established. This status quo is not only reflected in educational practice, but also reflects that the basic teaching objectives of the design are not strong and the structure of teachers is unreasonable. At the same time, it also reflects the backward teaching concepts and outdated teaching methods. It is reflected in the society that the students' comprehensive quality, sustainable development ability, and career extension space cannot meet the needs of the design market.

The basic courses under the systematic mode of disciplines are not suitable for the rapid development of the current information society. This kind of malady has become one of the chronic diseases that hinder the development of design education in colleges and universities. The teaching of basic courses for design majors in colleges and universities must be reformed. The depth of its reform and the number of achievements are important criteria to test and measure the quality of design education in colleges and universities. This has become the consensus of people in the contemporary design vocational education industry.

#### 3.2.4. Weak Practical Ability of Full-Time Teachers

Some teachers' professional theoretical knowledge is outdated. Although some teachers have a certain knowledge base, most teachers stay in the school to work directly and have no experience in designing companies. Therefore, professional practice teaching is a weakness, and teachers are unfamiliar with the specific knowledge of love mirrors. Teachers in the school lack the update and understanding of knowledge. They will not fully realize the importance of these practical skills in the cultivation of students' overall quality. Most teachers avoid the important in teaching, and the course is mainly theory. Due to the reduction of the practical teaching part, the graduates cannot achieve the goal of cultivating “practical” talents. The vast majority of teachers have not systematically studied design pedagogy and teaching theory and other related knowledge. It lacks sufficient understanding of the characteristics, laws, and professional teaching methods of design education. Therefore, it is impossible to provide effective design education guidance to students in teaching.

### 3.3. Current Situation of the Curriculum System of Environmental Design

#### 3.3.1. Single Course Mode

China's education system reform is constantly advancing, and environmental design education is no exception. Compared with foreign countries, this discipline in China starts relatively late. The curriculum education model still adopts the traditional public system, so the school-running features lack distinctiveness and the curriculum model is single. The talent training model is also relatively rigid and lacks innovation. It is difficult to make substantial progress if it is limited to a simple teaching and lecturing mode [17].

#### 3.3.2. Inadequate Teaching Facilities

The teaching facilities of some colleges and universities are relatively old and lack multimedia teaching equipment. At the same time, the hardware facilities cannot keep up, which may lead to a great reduction in the teaching level.

#### 3.3.3. Teaching Methods Are in Urgent Need of Innovation

Nowadays, the teaching method of most colleges and universities is still based on one-way teaching by teachers, and students are in a passive accepting position in learning. In this way, the teaching ability of teachers cannot be improved, and the teaching method is single. At the same time, students cannot participate effectively, which reduces students' interest and thinking and practical ability. There is less interaction with students, which will lead to students not being in the main position of the whole teaching process. Under the guidance of inherent thinking, most teachers teach in a one-way teaching method. And students have long been accustomed to passive acceptance. Over time, students will not only lose their ability to think independently, but also lose their interest in exploring and learning [18].

#### 3.3.4. The Structure of the Teaching Staff Needs to Be Improved

Teachers' own understanding of knowledge is not thorough enough. They cannot extend the knowledge they impart. At the same time, the teaching method itself has many shortcomings. Because the teaching team is too young, it has caused a lot of instability, and the mobility and loss of personnel are relatively large. However, senior teachers are too rigid in the traditional teaching model. It is difficult for such teachers to make great breakthroughs and improvements in teaching. As a result, there is a lack of a relaxed classroom atmosphere during the class. Therefore, the balance and perfection of the teaching staff are very important.

#### 3.3.5. The Quality of Teaching Needs to Be Improved

Colleges and universities blindly expand the scale of running schools and recruit a large number of students, and it is easy to ignore the improvement of teaching quality. Schools place too much emphasis on the acquisition of teaching benefits. The teaching quality of environmental design major needs to be improved.

#### 3.3.6. Students' Foundation Is Not Solid

In the environment of exam-oriented education, many students only take exams for their studies. Many students blindly choose majors and schools without a solid foundation, and they are even more blind in their future career choices. This creates a vicious circle. Later education and teaching are naturally more difficult to advance.

## 4. Construction and Application of the Curriculum System for Design Major

### 4.1. The Value of Curriculum Objectives in the Curriculum System

In the field of curriculum research, the study of curriculum objectives and their theories is an independent and very important part. In the course of constructing the curriculum system, the role of curriculum objectives is self-evident. In the circulatory system of curriculum system elements, curriculum objectives are both the starting point and the ending point. It is the directional guide of the whole curriculum system. It is the most basic and important principle to be followed in course setting. It is also the final direction of the other four elements of the curriculum system [19, 20].

The training goal of the integrated design major is the starting point for the construction of the design major curriculum system. It is necessary to consider the specific social environment or context and the background of big data environmental protection, and the four elements and links of the curriculum system can be successfully implemented. And when the course objectives are set, the expected results can be achieved. The course goal of design major is the orientation of design talents and the design coordinates of future development, and it is also an important lever for course adjustment. It plays a significant role in the breadth and depth of curriculum setting and the proportion of curriculum structure.

### 4.2. Specific Measures to Design Professional Curriculum Goals

#### 4.2.1. From Emphasizing “Double Base” to Emphasizing “Four Dimensions”

One of the important contents of “integration of industrialization and industrialization” is informatization. In a sense, the informatization of each element of the curriculum system also means the educational values of contemporary society and the value orientation of the curriculum system, which are directly reflected through the curriculum goals. Referring to the relevant literature on curriculum learning objectives at home and abroad, this paper believes that it is more appropriate to divide the curriculum objectives of industrial design education for “integration of industrialization and industrialization” into knowledge, skills, attitudes, and methods. At the same time, it should be supplemented by three levels of behavioral goals, generating goals, and expressing goals. It can also promote the multidimensional growth and development of students.

#### 4.2.2. Emphasis on “Information Literacy”

“Information literacy” requires the ability and attitude of “people” in contemporary society. It can be achieved through the representation of “information education class” and “wide use of information technology.” But the system theory point of view proves that the power of the whole system can solve the corresponding problem. The cultivation of “information literacy” can not only rely on the setting of courses, nor is it limited to the operation of technical means. These concepts should be infiltrated in the reform of the entire curriculum system. Facing the changes of society, the way of “responding to all changes with the same” is lagging behind. The goal of the course is to make a timely response to the era of “integration of industrialization and industrialization.” It can also be said to promote the transfer of curriculum values. However, this change is not a specific adjustment to the subject curriculum. It should be the overall and comprehensive penetration of the design curriculum system goals.

#### 4.2.3. Design Professional Talent Competency Framework

Environmental design mainly relies on environmental engineering and design. It is also an interdisciplinary and comprehensive marginal subject. The characteristics of environmental design discipline are also applicable to design education. At present, the state has put forward the strategy of “integration of industrialization and industrialization.” Under the background of the integration of informatization and industrialization, it is particularly important to integrate environmental design professionals with complex, innovative, applied, and diversified integration. Therefore, environmental design talents need to have various professional abilities such as integration and innovation for the social trend of “integration of industrialization and industrialization.” The increasingly complex design issues of the twenty-first century have involved all aspects of people, nature, and society in a globalized world. Many factors that affect the success or failure of a curriculum system are outside the internal elements. Therefore, the design curriculum system should also pay attention to external elements such as society and environment, humanities and ethics, teamwork, communication, and interdisciplinary in the design background. When a balance of internal and external elements is achieved, the curriculum system can prepare design graduates for industrial work.

### 4.3. Selection of Course Content for Design Majors

#### 4.3.1. The Value of Course Content in the Curriculum System

One of the most important research topics in the field of curriculum theory is the specific content of the curriculum. The content of the curriculum has a very important influence on the characteristics and abilities of talents. The content of the course reflects and realizes the goal of the course, and the function of the course must depend on the content of the course to be brought into play. Course content is the main basis for distinguishing industrial design majors from other majors. Course content is of great significance to the curriculum system. In fact, the process of selecting course content is not simply the questioning and selection of knowledge. It also reflects the deep content of teaching philosophy, values and so on.

### 4.4. Specific Measures to Design Professional Course Content

The knowledge structure contains many elements, and it presents multiple levels. When these elements are combined in a reasonable way, they can work best by themselves. Under the background of “integration of industrialization and industrialization,” the knowledge structure of design talents should show the characteristics of fonts, and there should be different levels within it. The author has established a pyramid-like knowledge system of environmental design talents in the context of “integration of industrialization and industrialization,” as shown in Figure 5. This model shows that under the background of “integration of industrialization and industrialization,” environmental design talents should have profound knowledge and high professionalism at the same time. The pyramid-like structure is conducive to the subject's open mind. It can also enable the subject to use professional thinking and professional knowledge to think about problems and propose creative solutions. At the same time, it can learn from the knowledge of other disciplines and obtain innovative inspiration. This is conducive to discovering new fields from the intersection of disciplines and innovating in this field.

The course content should cover the knowledge of this major and adjacent majors. The course content not only imparts theory and knowledge to students, but also focuses on cultivating and exercising students' abilities and qualities. The course content should pay attention to cultivating and improving students' cultural literacy, and should focus on cultivating students' learning ability, practical ability, and innovative thinking. Students should be encouraged to explore and research independently, and organically combine quality education and ability education.

### 4.5. Integration of Environmental Protection and Big Data with Course Content

The course content for the “integration of industrialization and industrialization” needs to pay more attention to the nature of environmental protection and big data design. Environmental protection design is a synthesis of environmental science and art, but it is fundamentally different from the nature of design and science. Scientific activities are centered on invention, while technological activities are centered on discovery. Environmental design activities are based on creation. Design pursues innovation and is constantly changing. Especially in the context of today's big data, the process of design pursuit of innovation is also a dynamic process. But the kernel of the environment design never changes. The core of this is that design is an environmental protection activity that humans consciously carry out in order to achieve a certain purpose. It is future-proof and also innovative. Design thinking is also different from artistic and scientific thinking. It is a thinking that integrates analysis, divergence, synthesis, diversity, innovation, and differentiation. The distinguishing feature of today's society is the knowledge economy. This puts forward higher requirements for the innovation of environmental design. The so-called design is essentially the rearrangement of the knowledge structure. It is also to reintegrate the existing resources and innovate the industrial mechanism. By enabling human beings to achieve sustainable development, it can meet the overall requirements of human survival and development.

### 4.6. Addition of Science and Technology Frontier Courses

With the rapid development of science and technology, not only science and technology are constantly being updated, but also scientific concepts are being updated. Therefore, in order to conform to the development of the times, Chinese environmental design has correspondingly added content related to modernization in its curriculum. From the perspective of the long-term development of environmental design, there must be courses related to the development of science and technology in teaching the activities of design. Through the opening of this course, students can master the new trends of scientific and technological development in today's world. At the same time, it can master certain advanced science and technology. It can also be applied to its design. Through the advancement of science and technology, the problems encountered in the design are solved. It is beneficial to improve the scientificity and practicability of the design or product.

### 4.7. Open Information Technology Courses

In educational activities for environmental design, courses related to information development should be offered. Through the teaching of the course content, students can improve their ability to collect and use scientific and technological information. Possessing this ability is to prepare students for the needs of an evolving society. The development of Internet information technology has raised the requirements for environmental design students to a certain extent. It must have the corresponding modern information to deal with the development of information technology.

Informatization talents have different training methods in different fields, and their roles are not the same. But there is one thing in common, while expanding the horizon of talent information, talent informatization can be used as a means to promote communication between talents in different fields. In turn, different disciplines can learn from each other and complement each other.

### 4.8. Structural Idea

The concept of curriculum structure needs to have the following three aspects of thinking.

#### 4.8.1. Clarifying the Goal, Building a Framework, Waiting for the Opportunity, and Improving the Practice

During the student period, the main goal of teaching is to help students complete a period of growth from professional enlightenment to entry. Although the previous series of studies have been fruitful, the details of the teaching content under the new teaching idea are still preliminary. It is necessary to design a curriculum structure framework according to the requirements of integrating big data and environmental protection. It is expected that under this framework, the ideas can be verified through teaching practice. And the specific content and connotation of each course can be enriched and improved.

#### 4.8.2. In-Depth Study and Comprehensive Application

Deep learning requires ample study time and coherence. The learning time span of each professional skill is no less than one year. The dominant idea is to emphasize the in-depth study of various software, scientific knowledge, and their synergistic applications. Integrated application refers to the overall link between course content. On the basis of in-depth study, comprehensively apply the acquired knowledge and skills through teaching-based design projects and practical work tasks in enterprises. Applying knowledge can be the focus of studio teaching and the inherent needs of students to complete their studies.

#### 4.8.3. Proportion of Professional Class Hours

Now, the respective proportions of professional courses and public culture courses in the total class hours of a school with environmental art design from 2018 to 2021 are calculated. The statistical results are shown in Figure 6.

Each professional course and each public culture course were broken up separately during the course arrangement and interspersed with each other in the class schedule. Cultural courses and professional courses are given equal attention, and the courses are arranged centrally. It needs to ensure the integrity and coherence of professional teaching. The specific schedule can be seen in Table 1.

### 4.9. Course Evaluation

#### 4.9.1. Professional Basic Assessment

It is stipulated that after completing the professional basic courses in the first academic year, students must participate in a professional basic skills assessment organized by the school's professional department. Students who fail to pass the examination will be treated as repeating grades. If it can be implemented, it will definitely cause the necessary learning pressure to the students. It can better ensure the starting point requirements of studio project teaching.

#### 4.9.2. Work Evaluation Mechanism

It is necessary to weaken the traditional mid-term and final examination assessment mode and strengthen the work practice evaluation orientation. A work practice evaluation mechanism can be established. It is stipulated that at the end of each semester, each student studio team must submit a work practice report and design work. All teachers are organized by the professional department. It needs to focus on reviews and ratings. This will be considered the grade for the semester.

#### 4.9.3. Enterprise Evaluation Mechanism

Studio logs and monthly schedules need to be created for each studio. It is necessary to count and sort out the work output of each studio on a monthly basis. Business feedback needs to be collected on a regular basis. There is a need to develop a corporate feedback response mechanism for the studio. Formulating an appropriate studio incentive and reward system can not only actively interact with the enterprise, but also enrich the form and connotation of the enterprise evaluation mechanism.

#### 4.9.4. Graduation Design Evaluation Mechanism

The content of graduation design includes three parts: research, graduation design creation, and production practice, which run through the entire student period. The final presentation form is to organize a student graduation project report exhibition every year. This exhibition can be regarded as a comprehensive report of the students' three-year professional learning results. It is the basis for our evaluation of students, and it is also a centralized review of the teaching effect. The establishment and improvement of the graduation design system are of great significance for improving the teaching process, evaluating the teaching quality, and accumulating teaching materials.

## 5. Analysis of Fuzzy Comprehensive Evaluation Effect

Big data provides a reference for the construction and application of the design major curriculum system. The third chapter constructs the curriculum system of design major. However, whether the constructed curriculum system of design major is scientific and reasonable needs to be evaluated. Due to the influence of multiple factors, the evaluation cannot be quantitatively evaluated. The author introduced the fuzzy comprehensive evaluation method in this research. This method is a comprehensive evaluation method based on fuzzy mathematics. It can effectively transform qualitative evaluation into quantitative evaluation [21–23]. Therefore, the problem of systematic evaluation of the fuzzy and difficult to quantify factors in the evaluation process can be solved.

### 5.1. Selecting Judgment Objects and Scope

This study will evaluate the quality and effect of the curriculum system of design majors under the environment of integrating environmental protection and big data. The object and scope of the evaluation are school teachers majoring in design.

### 5.2. Establishing and Determining the Index Set *U* of the Evaluation Object

Through the review of relevant literature, the rules and elements of the fuzzy comprehensive evaluation method are sorted out. Combined with the practical investigation of the evaluation system of classroom teaching mode, this research determines that the index set of the evaluation object is *U*. It includes four levels: teaching environment (*A*), classroom response (*B*), teacher satisfaction (*C*), and teaching effect (*D*). The specific indicators can be expressed as follows.

The teaching environment includes the degree of informatization environment construction (A1), the degree of intelligence of the teaching process (A2), and the ease of operation of the equipment system (A3). Classroom responses include students' overall attitude towards learning (B1), students' enthusiasm for learning (B2), improvement of collaboration and communication skills (B3), application of innovative mechanisms (B4), and rationality of the setting of wisdom links (B5). Teacher satisfaction includes the satisfaction of classroom students' learning status (C1), the reform and innovation of the professional curriculum system (C2), the psychological changes of students' acceptance of the system (C3), and the comparison of teaching effects before and after the application of the system (C4). The teaching effect includes a firm grasp of students' basic knowledge and theory, improvement of students' ability to analyze and solve problems, active classroom atmosphere, active cooperation of students, and achievement of teachers' teaching and students' abilities.

### 5.3. Constructing the Judgment Matrix Corresponding to Each Level

In order to construct the judgment matrix corresponding to each level and determine the corresponding evaluation index weight, the 1–9 scaling method is introduced, as shown in Table 2 [24, 25].

According to the construction of the above indicators and the statistics of relevant questionnaire data, the first-level indicators and the second-level indicators are compared. After comparing the two indicators, a set of judgment matrices (represented by *U*, *A*, *B*, *C*, *D* respectively) are obtained as follows:

(1) $$\begin{array}{c} U=\left[\begin{array}{cccc} 1 & \frac{1}{3} & \frac{1}{3} & \frac{1}{5}\\ 3 & 1 & 1 & \frac{1}{2}\\ 3 & 1 & 1 & \frac{1}{2}\\ 5 & 2 & 2 & 1 \end{array}\right],\\ A=\left[\begin{array}{ccc} 1 & \frac{1}{3} & 3\\ 3 & 1 & \frac{1}{2}\\ \frac{1}{3} & 2 & 1 \end{array}\right],\\ B=\left[\begin{array}{ccccc} 1 & \frac{1}{3} & \frac{1}{2} & 1 & \frac{1}{4}\\ 3 & 1 & 1 & 2 & \frac{1}{2}\\ 2 & 1 & 1 & 2 & \frac{1}{2}\\ 1 & \frac{1}{2} & \frac{1}{2} & 1 & \frac{1}{4}\\ 4 & 2 & 2 & 4 & 1 \end{array}\right],\\ C=\left[\begin{array}{cccc} 1 & 2 & 2 & \frac{1}{3}\\ \frac{1}{2} & 1 & 1 & \frac{1}{3}\\ \frac{1}{2} & 1 & 1 & \frac{1}{3}\\ 1 & 3 & 3 & 1 \end{array}\right],\\ D=\left[\begin{array}{cccc} 1 & \frac{1}{6} & 2 & 1\\ 6 & 1 & 7 & 2\\ \frac{1}{2} & \frac{1}{7} & 1 & \frac{1}{2}\\ 1 & \frac{1}{2} & 2 & 1 \end{array}\right]. \end{array}$$

Due to the pairwise comparison of the various factors involved in the effect application evaluation, there may be conflicting situations, and it is impossible to make a completely correct judgment. In the course of the research, almost all pairwise comparisons are allowed to have some degree of inconsistency. To solve this problem, a consistency check is required. The maximum eigenvalues of each matrix are calculated as *λ*_*A*_ = 3.038, *λ*_*B*_ = 5.0198, *λ*_*C*_ = 4.0501, and *λ*_*D*_ = 4.1153.

In order to determine the allowable range of the degree of inconsistency, the corresponding average random consistency index RI value is found according to the requirements. The RI values are shown in Table 3.

The calculation formula of the consistency index is as follows:

(2) $$\begin{array}{c} \text{CI}=\frac{\lambda_{\max}-n}{n-1},\\ \text{CR}=\frac{\text{CI}}{\text{RI}}, \end{array}$$

where *λ*_max_ is the largest eigenroot of the judgment matrix.

The calculated consistency indicators are CR_*A*_ = 0.0327, CR_*B*_ = 0.0044, CR_*C*_ = 0.0185, and CR_*D*_ = 0.0427. The CR results obtained were all less than 0.1. Therefore, the judgment matrices have good consistency. The relative weight vector of indicators at all levels is calculated by the summation method. The eigenvector value corresponding to each level factor is *Y*.

(3) $$\begin{array}{c} Y_{U}=\left[\begin{array}{c} 0.082\\ 0.235\\ 0.235\\ 0.448 \end{array}\right],\\ Y_{A}=\left[\begin{array}{c} 0.332\\ 0.361\\ 0.286 \end{array}\right],\\ Y_{B}=\left[\begin{array}{c} 0.092\\ 0.216\\ 0.198\\ 0.099\\ 0.395 \end{array}\right],\\ Y_{C}=\left[\begin{array}{c} 0.235\\ 0.138\\ 0.138\\ 0.489 \end{array}\right],\\ Y_{D}=\left[\begin{array}{c} 0.150\\ 0.572\\ 0.083\\ 0.196 \end{array}\right]. \end{array}$$

Through the online distribution and recycling of the evaluation questionnaire on the effect of this model, the comprehensive evaluation of 16 experts or teachers is collected. The statistical results are shown in Figure 7.

The change law of the four evaluation levels is shown in Figure 8.

By summarizing the process of experts participating in the evaluation and combining with the questionnaire, four evaluations are carried out on the 16 indicators. After data statistics and sorting, the corresponding fuzzy evaluation moments are obtained.

(4) $$\begin{array}{c} R1=\frac{1}{16}\left[\begin{array}{cccc} 3 & 7 & 6 & 0\\ 4 & 6 & 6 & 0\\ 4 & 8 & 4 & 0 \end{array}\right],\\ R2=\frac{1}{16}\left[\begin{array}{cccc} 7 & 5 & 4 & 0\\ 9 & 6 & 1 & 0\\ 6 & 8 & 2 & 0\\ 8 & 6 & 2 & 0\\ 7 & 8 & 1 & 0 \end{array}\right],\\ R3=\left[\begin{array}{cccc} 6 & 7 & 3 & 0\\ 7 & 5 & 4 & 0\\ 6 & 8 & 2 & 0\\ 9 & 5 & 2 & 0 \end{array}\right],\\ R4=\left[\begin{array}{cccc} 8 & 6 & 2 & 0\\ 5 & 8 & 3 & 0\\ 7 & 7 & 2 & 0\\ 6 & 7 & 3 & 0 \end{array}\right]. \end{array}$$

The evaluation result set in four aspects of teaching environment, classroom response, teacher satisfaction, and teaching effect can be calculated as follows:

(5) $$\begin{array}{c} \left\{\begin{array}{c} R1=\left[\begin{array}{cc} 0.224 & 0.424\;0.331\;0 \end{array}\right],\\ R2=\left[\begin{array}{cc} 0.458 & 0.443\;0.098\;0 \end{array}\right],\\ R3=\left[\begin{array}{cc} 0.475 & 0.368\;0.157\;0 \end{array}\right],\\ R4=\left[\begin{array}{cc} 0.364 & 0.464\;0.173\;0 \end{array}\right]. \end{array}\right) \end{array}$$

After normalizing the result set, *R*′ can be obtained:

(6) $$\begin{array}{c} R{}^{\prime }=\left[\begin{array}{cccc} 0.229 & 0.433 & 0.338 & 0\\ 0.459 & 0.443 & 0.098 & 0\\ 0.475 & 0.368 & 0.157 & 0\\ 0.364 & 0.463 & 0.173 & 0 \end{array}\right], \end{array}$$

Through the comprehensive evaluation of two levels, the evaluation result set is finally obtained:

(7) $$\begin{array}{c} R=\left[\begin{array}{cccc} 0.401 & 0.434 & 0.165 & 0 \end{array}\right], \end{array}$$

The comprehensive evaluation set is set as *V* = {excellent, good, fair, poor}, and the corresponding scores are shown in Table 4.

A corresponding score needs to be set for each evaluation level. It can be set to 95, 75, 55, 25, respectively. The evaluation level parameter matrix is *V*′ = {95, 75, 55, 25}. The evaluation result *S* is

(8) $$\begin{array}{c} S=\left[\begin{array}{cccc} 0.401 & 0.434 & 0.165 & 0 \end{array}\right]\left[\begin{array}{c} 95\\ 75\\ 55\\ 25 \end{array}\right]=79.72>60. \end{array}$$

The evaluation result is good on the upper side. By using the fuzzy comprehensive evaluation method, the author conducts a comprehensive analysis and evaluation of the construction and application of the curriculum system of the design major under the environment of big data and environmental protection. The final comprehensive application effect is good. It is fully proved that the application of this model to teaching is beneficial to enhance students' perception of the classroom. It is beneficial to improve students' classroom enthusiasm and interaction, to improve students' collaboration and communication ability, to improve students' ability to analyze and solve problems, to improve classroom teaching efficiency, and to promote the generation of teachers' teaching and students' learning ability, etc.

### 5.4. Evaluation Effect Feedback

Based on big data and environmental protection, the construction of professional curriculum system needs to be designed in detail. The system is also applied to the classroom of specific subject teaching. In the later period, the author collected valuable opinions and survey feedback from experts and teachers on this system by using the survey method and interview method. Then, various evaluation indicators are designed. The comprehensive effect of applying this model in the classroom is judged. It is known from the results that the effect of applying this model is good. It shows that this model has brought spring for the innovation of teaching model and the development of education informatization. But there is still room for further improvement. In the subsequent use process, the teaching process in this mode can also be optimized and improved to provide a more efficient and smarter classroom teaching mode for education and teaching.

## 6. Conclusion

The fact that the curriculum is oriented towards the “integration of industrialization and industrialization” does not mean from the “traditional industrialization” side of the pendulum. It can be completely swayed to the other end of “informatization.” Instead, it seeks to balance the fulcrum of theory and practice, and achieve connection, transformation, and transcendence in dynamic adjustment. The “integration of industrialization and industrialization” in reality does not mean abandoning the “design based on scientific and technological knowledge” that was emphasized in the past. It is to emphasize that industrial design education should be in line with “informatization.”

The comprehensive application effect of this model is evaluated and analyzed by the fuzzy comprehensive analysis method. The factors affecting the teaching effect after the implementation of this model are investigated and analyzed first. By adopting the valuable opinions of experts and teachers, a set of relevant indicators was designed and the effectiveness of the indicators is verified. The conclusion is drawn that the classroom teaching effect is good after applying this model. Finally, the questionnaire survey method and fuzzy comprehensive evaluation method are used to verify the good application effect of this model. The validity of this model is further verified.

The optimization of curriculum structure is the focus of school-level curriculum reconstruction. The direction of optimizing the curriculum structure of environmental design education in China should focus on adjusting the integration of general education and professional courses in the curriculum structure. At the same time, attention should be paid to the integration and integration of subject courses, the modularization of compulsory and elective courses, the integration of theoretical courses and practical courses, and the synergy of explicit and implicit courses. The “modular curriculum structure model” of China's environmental design major proposed in this study can be used as a reference for the reform of the curriculum system of environmental design education in colleges and universities.

## Figures and Tables

**Figure 1:** Changes in the number of design colleges and graduates in the past ten years. (a) Number of graduates and colleges. (b) Practitioners as a percentage of the number of graduates that year.

**Figure 2:** Advantage feature map.

**Figure 3:** Curriculum system elements.

**Figure 4:** The relationship between the ability of the above survey results and the proportion of supporters.

**Figure 5:** “Integration of informatization and industrialization” design talent knowledge system.

**Figure 6:** The respective proportions of professional courses and public culture courses in the total class hours. (a) Class. (b) Proportion.

**Figure 7:** The statistical results. (a) First-level indicator. (b) Secondary indicators.

**Figure 8:** The change law of the four evaluation levels.

**Table 1:** Suggested schedule for design majors.

Section number		Sunday	Monday	Tuesday	Wednesday	Thursday	Friday
Morning	Section 1	Holiday	Professional course	Professional course	Professional course	Professional course	Cultural course
	Section 2						
	Section 3						
	Section 4						

Afternoon	Section 5	Holiday	Cultural course	Cultural course	Cultural course	Cultural course	Cultural course
	Section 6						

Evening study	Section 7	Professional course	Professional course	Professional course	Cultural tutoring	Cultural tutoring	Holiday
	Section 8						

**Table 2:** 1–9 scale.

Relative importance level setting	Meaning description
1	Equally important
3	Slightly important
5	Obviously important
7	Strongly important
9	Extremely important
1/3	Slightly unimportant
1/5	Obviously unimportant
1/7	Strongly unimportant
1/9	Extremely unimportant
2, 4, 6, 8, 1/2, 1/4, 1/6, 1/8	The importance is between the two adjacent levels above

**Table 3:** Values of the average random consistency index RI.

*n*	1	2	3	4	5	6	7	8	9
RI	0	0	0.58	0.9	1.12	1.24	1.32	1.41	1.45

**Table 4:** Corresponding score table of comprehensive evaluation.

Rank	Excellent	Good	Generally	Poor
Score	[80, 100]	[60, 80]	[40, 60]	[0, 40]

## Data Availability

The dataset can be accessed upon request.
